# The Value of Color Doppler Ultrasound and CT Combined with Serum AFP Examination in the Diagnosis of Hepatocellular Carcinoma

**DOI:** 10.1155/2022/4147753

**Published:** 2022-03-26

**Authors:** Peiwan Jia, Yunjie Mao, Kahua Liu, XianJuan Wei

**Affiliations:** ^1^Department of Imaging, Jiaozhou Central Hospital, Qingdao 266300, China; ^2^Anorectal Department, Rizhao Hospital of TCM, Rizhao 276800, China; ^3^Department of Gastroenterology, The Affiliated Qingdao Central Hospital of Qingdao University, The Second Affiliated Hospital of Medical College of Qingdao University, Qingdao 266042, Shandong, China; ^4^Department of General Surgery (I), Qingdao Hospital of Traditional Chinese Medicine, Qingdao Hiser Hospital Affiliated to Qingdao University, Qingdao 266033, China

## Abstract

**Objective:**

To evaluate the value of the combination of color Doppler ultrasound, computed tomography (CT), and serum tumor marker alpha-fetoprotein (AFP) examination in the diagnosis of hepatocellular carcinoma (HCC).

**Methods:**

98 patients with HCC (malignant tumor group) and 50 liver lesion patients (benign control group), were selected for the study, and retrospective statistical methods were used to evaluate the diagnostic values of the three examinations on hepatocellular carcinoma.

**Results:**

(1) When comparing color Doppler ultrasound blood flow parameters, the hepatic artery diameter, peak flow velocity, minimum flow velocity, and resistance index (RI) of hepatocellular carcinoma were significantly higher than those of the benign control group (*P* < 0.05), while the portal vein flow velocity was significantly lower than that of the control group (*P* < 0.05). (2) Enhanced CT imaging of hepatocellular carcinoma lesions showed mostly outflow-type enhancement changes, with high- or slightly high-density shadowing and uneven enhancement in the arterial phase, relatively low density and withdrawal of enhancement in the portal vein phase and delayed phase. (3) The serum AFP level of hepatocellular carcinoma patients was significantly higher than that of the benign control group (*P* < 0.01). (4) The sensitivity of color Doppler ultrasound, CT, and serum AFP alone for the diagnosis of HCC was 79.59%, 85.71%, and 66.33%, and the accuracy was 83.78%, 87.16%, and 74.32%, respectively, while the combination of the three tests could significantly increase the sensitivity to 96.94% and the accuracy to 93.92%, compared with each individual test (*P* < 0.01).

**Conclusion:**

Color Doppler ultrasound and CT combined with serum AFP examination could significantly improve the sensitivity and accuracy of hepatocellular carcinoma diagnosis, reduce misdiagnosis, and facilitate early diagnosis and clinical early intervention.

## 1. Introduction

Primary liver cancer (PLC) is a malignant tumor that originates in the liver and is currently the sixth most common cancer in the world, ranking fourth in cancer-related deaths, with hepatocellular carcinoma (HCC) accounting for more than 85%–90% of these cases, posing a serious threat to human health [1]. In recent years, the incidence of hepatocellular carcinoma has been increasing year by year with the increase of life stress, frequent food safety incidents, and increasingly serious environmental pollution caused by industrialization [2]. At present, surgical resection, liver transplantation, and intervention are the main effective methods to treat early HCC, but there are no specific symptoms in the early stage of the disease, and most patients are already in the middle and late stages when they are diagnosed, thus losing the best treatment opportunity, resulting in poor prognosis and high mortality [3]. Liver tissue aspiration pathological biopsy is standard for primary liver cancer diagnosis, but it is an invasive test and not suitable for screening, early diagnosis, and prognostic follow-up of high-risk groups [4]. At present, screening and early diagnosis of HCC still mainly rely on serology and imaging. Alpha-fetoprotein (AFP) was once the most classic marker for the diagnosis of HCC, but about 20%–30% of HCC patients had negative or low AFP expression [5]; for imaging screening, color Doppler ultrasound is currently the most widely used imaging screening tool because of its noninvasive and convenient nature, but ultrasonography may be affected by rib obscuration, abdominal wall, intestinal gas, and other factors that may lead to misdiagnosis imaging [6]. Currently, with the development of imaging medicine, intensive CT has become one of the main examination methods for diagnosing hepatocellular carcinoma, but it also has some limitations.

## 2. Materials and Methods

### 2.1. Clinical Materials

Clinicopathological data of 98 patients with HCC first diagnosed in our hospital between January 2017 and December 2019 were collected consecutively. Gender: 59 males and 39 females; age 35–81 years, mean (57.32 ± 6.81) years; clinical stage: stage I (18 cases), stage II (47 cases), stage III (24 cases), and stage IV (9 cases); degree of differentiation: 37 cases of highly differentiated, 26 cases of moderately differentiated, 20 cases of lowly differentiated, and 15 cases of undifferentiated. Inclusion criteria are as follows: (i) 98 patients with HCC were diagnosed by pathological histology; (ii) all were single lesions and were not treated with radiotherapy before hospitalization; (iii) all had color Doppler ultrasound, CT, and serum AFP examination data before treatment. Exclusion criteria are as follows: (i) metastatic liver cancer; (ii) incomplete study data; (iii) with other malignant tumors; and (iv) with other chronic liver diseases. Fifty patients with benign liver lesions attending the same period were selected as benign controls, 5 cases of hepatitis pseudotumor, 9 cases of hepatic hemangioma, 23 cases of cirrhotic hyperplastic nodules, and 13 cases of hepatic granuloma. Sex: 32 males and 18 females; age: 33–85 years, mean (55.67 ± 8.42) years. Inclusion criteria are as follows: (i) all had color Doppler ultrasound, CT, and AFP examination data; and (ii) all had benign liver lesions. There was no statistical difference between the two groups in terms of baseline information such as gender and age (*P* > 0.05), and they were comparable (Table 1). The study was approved by the ethics committee of our hospital (ethics approval number: LUNLIHao: 2018010), and informed consents were signed with the study subjects to participate in the study voluntarily.

### 2.2. Color Doppler Ultrasonography

The diagnostic instrument was a PHILIPS iU22 with a probe frequency of 3.5–5.0 MHz. The patient was placed in a supine position with a morning fast of more than 8 hours and was carefully scanned by a physician specialized in ultrasound for all sections of the liver. The size and morphology of the liver were firstly observed, and then the location, size, morphology, and boundary of the mass and the internal echo of the lesion were carefully observed. Subsequently, the blood supply and blood flow inside and around the tumor were observed using the color ultrasound mode. The blood flow parameters such as hepatic artery diameter (mm), peak hepatic artery flow velocity (cm/s), minimum hepatic artery flow velocity (cm/s), portal vein flow velocity (cm/s), and resistance index (RI) were also measured with the help of PW mode. Each patient was measured 3 times, and the mean value was taken.

### 2.3. CT Examination

The instrument was a Siemens 64-slice CT scanner, and the patient was placed in a supine position. During the examination, the patient was instructed to keep the upper arm in an upward position and to hold breath, and the scanning area was the upper abdomen. The tube voltage was 120 kV, the layer spacing was set at 5 mm, and the layer thickness was 5 mm. The upper abdomen was scanned first, and then, 100 mL of iohexol was injected through the elbow vein at a flow rate of 3 mL/s, and the scan was performed in the arterial phase (30s), portal phase (60–70s), and delayed phase (120–180s). The number of lesions, density, boundary, and dynamic enhancement scan characteristics and enhancement exit features were observed.

### 2.4. Serum AFP Examination

4 ml of venous blood was drawn from each of the malignant tumor group and benign control group on an empty stomach at 6.00–9.00 a.m., and the serum was separated for examination by centrifugation after standing for self-coagulation. AFP was detected by electrochemiluminescence using the German Roche E601 automatic immunoassay analyzer; the procedure was carried out strictly according to the operating instructions. Normal reference value: AFP<20 ng/ml.

### 2.5. Determination of Results

The ultrasound and CT examination results of the liver cancer group were true positive if they were consistent with the pathological diagnosis, and false negative if they were inconsistent with pathological diagnosis as the gold standard. The results of ultrasound and CT in the benign control group were true negative and false positive when they were inconsistent with pathological diagnosis. Serum AFP levels above the threshold were considered positive and at or below the threshold were considered negative. If there were one or more positive items in the combined test, it shall be regarded as positive; all negative was defined as negative.

### 2.6. Statistical Analysis

SPSS22.0 statistical software was used for data analysis and processing. Mean ± standard deviation (‾*x* ± *s*) was used to describe the concentration levels of measurement data, and an unpaired *t*-test was used for comparison between the two groups. The count data were expressed as a rate (%), and the comparison between groups was performed by *χ*^2^ test. The value of ultrasonography, CT, and AFP alone and combined in the diagnosis of hepatocellular carcinoma was statistically calculated by four grids with pathological diagnosis as the standards. The test diagnostic results were divided into true positive (a), false positive (b), false negative (c), and true negative (d). *P* < 0.05 was considered statistically significant.

## 3. Results

### 3.1. Comparison of Serum AFP Levels between the HCC Group and Benign Control Group

The serum AFP level in the hepatocellular carcinoma group was (159.3232.49) ng/ml, the serum AFP level in the benign control group was (15.823.02) ng/ml, and the difference was statistically significant, *P* < 0.01.

### 3.2. Color Doppler Ultrasonography of Hepatocellular Carcinoma

The color Doppler ultrasonography of 98 patients with hepatocellular carcinoma accorded with the pathological diagnosis of 78 cases and inconsistent in 20 cases (including 6 lesions misdiagnosed as hepatitis pseudotumors, 4 misdiagnosed as hepatic hemangiomas, 7 misdiagnosed as cirrhotic hyperplastic nodules, and 3 misdiagnosed as hepatic granuloma). The color Doppler ultrasonography of 46 cases in the control group was consistent with the pathological diagnosis and inconsistent in 4 cases (4 cases were misdiagnosed as hepatocellular carcinoma).

The ultrasound images of hepatocellular carcinoma mostly showed regular or irregular morphology, and the internal echogenicity was mostly hypoechoic, but as the tumor enlarged larger lesions could be isoechoic, hyperechoic, or more strongly echogenic under ultrasound and accompanied by partial tissue liquefaction and necrosis. For comparison of blood flow parameters, the hepatic artery diameter, peak flow velocity, minimum flow velocity, and resistance index (RI) of hepatocellular carcinoma were significantly higher than those of benign controls (*P* < 0.05), and the portal vein flow velocity was significantly lower than that of controls (*P* < 0.05, Table 2). Color Doppler ultrasound sonography of HCC is shown in Figure 1.

### 3.3. Enhanced CT Image of Hepatocellular Carcinoma

Using a pathological diagnosis as the gold standard, the enhanced CT images of 84 patients (confirmed cases) with HCC accorded with the pathological diagnosis and 14 cases were inconsistent (5 cases of small hepatocellular carcinoma foci were missed, 2 cases were misdiagnosed as inflammatory pseudotumors, 5 cases were misdiagnosed as cirrhotic hyperplastic nodules, and 2 cases were misdiagnosed as hepatic hemangioma). The enhanced CT images of the control group accorded with pathology in 45 cases and inconsistent in 5 cases (5 cases were misdiagnosed as hepatocellular carcinoma).

Enhanced CT showed that most hepatocellular carcinoma lesions showed outflow-type intensification changes, with high- or slightly high-density shadow in the arterial phase and uneven intensification, and relatively low density in the portal vein phase and delayed phase, and the degree of intensification continued to decrease, showing “fast-revealing and fast emerging” intensification. The enhanced CT image of HCC is shown in Figure 2.

Comparison of the value of color Doppler ultrasound, CT, and AFP alone and in combination for the diagnosis of hepatocellular carcinoma.

The results of color Doppler ultrasound, CT, and serum AFP for the diagnosis of hepatocellular carcinoma were compared with the pathological diagnosis as the gold standard, as shown in Table 3. The values of color Doppler ultrasound, CT combined with serum AFP alone, and combined examination for the diagnosis of HCC were compared, as shown in Table 4. The sensitivity, accuracy, and negative predictive value of the combination examination were significantly improved compared with each examination, *p* < 0.01.

## 4. Discussion

Clinical treatment for mid-to late-stage primary liver cancer is poor and effective therapies are lacking; therefore, early diagnosis of hepatocellular carcinoma and clarification of the extent of its lesions are of great clinical value in guiding the establishment of treatment modalities. The diagnosis of hepatocellular carcinoma rarely relies on pathological puncture biopsy [6], and the National Comprehensive Cancer Network (NCCN) guidelines use alpha-fetoprotein (AFP) and upper abdominal ultrasound as diagnostic criteria for hepatocellular carcinoma. The guidelines recommend that patients with cirrhosis routinely undergo an abdominal ultrasound and serological tumor markers every 6 months to improve the detection rate of early hepatocellular carcinoma [7]. However, there are limitations in diagnosing hepatocellular carcinoma solely from serum AFP and ultrasonography.

AFP is a glycoprotein that is produced by the fetal liver and yolk sac during gestation and is present in low levels in the peripheral blood after birth. When hepatocellular carcinoma occurs, the AFP synthesis gene can be initiated in cancer cells to produce and secrete AFP [8]. AFP is the earliest marker for the diagnosis of hepatocellular carcinoma and is currently the preferred marker for laboratory screening of primary hepatocytes. The practice has confirmed that AFP can be used as an HCC diagnostic, efficacy evaluation, and prognostic assessment of laboratory indicators [9]. However, not all hepatocellular carcinoma cells secrete AFP, and there are still some patients with hepatocellular carcinoma with negative or low concentrations [5], and additional causes of elevated AFP can be seen in pregnancy and malignancies of gonadal origin [9]. Therefore, AFP testing alone has a certain rate of underdiagnosis for the prediction of hepatocellular carcinoma.

Color Doppler ultrasound diagnosis is a noninvasive, painless, convenient, and intuitive effective examination means, which can not only observe the morphology of the tumor but also can clearly and intuitively display the blood flow characteristics inside the HCC tumor and has a good detection of blood flow signal grading, blood supply artery, collateral circulation, and portal vein of the tumor [10]. HCC requires high blood supply, so according to the tumor tissue inside, the graded blood flow signal can reflect the aggressiveness of liver cancer tissue [11]. Abundant blood supply allows cancer cells to obtain conditions for rapid growth and metastasis, accelerating lesion progression [12]. Observation of hepatic artery diameter, peak flow rate, minimum flow rate, and resistance index (RI), and thus more visualization of blood flow in hepatocellular carcinoma tissues can help determine the degree of lesion progression [13]. However, some benign and malignant lesions are more difficult to identify.

In comparison, CT examination has high image resolution and is not interfered with by factors such as gas, obesity, and breathing and can display the anatomical structure of the human liver, which can realize multiangle, multidirectional, and multitemporal observation of lesion characteristics and can improve the accuracy of liver cancer diagnosis, while having its higher qualitative diagnostic advantage [14]. The liver is a dual blood supply organ, in which the hepatic artery blood supply accounts for 20% and the portal vein accounts for about 80%. Hepatocellular carcinoma is mainly supplied by the hepatic artery, and in the early stage of enhancement, the CT value rises significantly and exceeds the liver parenchyma, showing early high-density enhancement, but the peak residence time of the lesion is short, after which the CT value of the lesion decreases, while the liver parenchyma reaches its peak in the portal vein phase, and the lesion is relatively with low density, with a fast-in and fast-out type of time density [15]. CT enhancement scanning improves the detection rate of hepatocellular carcinoma lesions by observing the dynamic process of contrast circulation in the liver [16, 17], but there are deficiencies in all hepatocellular carcinoma lesions ≤3.0 cm in diameter, and clinical diagnosis requires attention [18].

Hepatocellular carcinoma is spatially and temporally heterogeneous, and invasive examinations cannot provide comprehensive information, so imaging plays a crucial role in the diagnosis of HCC. Noninvasive imaging can be the basis for diagnosis and treatment before the biopsy. Numerous liver cancer guidelines include multiphase CT/MRI scanning as important tools for the diagnosis and evaluation of HCC [19, 20]. The current study showed that color Doppler ultrasound, CT, and serum AFP could be used as diagnostic methods for hepatocellular carcinoma. However, the values of a single examination were limited, with sensitivities of 79.59%, 85.71%, and 66.33%, and accuracies of 83.78%, 87.16%, and 74.32%, respectively, which were far from meeting clinical diagnostic needs. The combined tests could complement each other and corroborate each other, which could effectively improve the sensitivity and accuracy of HCC diagnosis to 96.94% and 93.92%, respectively.

In conclusion, color Doppler ultrasound and CT combined with serum AFP examination for the diagnosis of HCC could significantly improve the diagnostic value of HCC.

## Figures and Tables

**Figure 1:** (a) Ultrasound two-dimensional image showed that the morphology of the liver section was abnormal, the volume was obviously increased, the surface of the liver capsule was not smooth, the intrahepatic echo was thickened and enhanced, the distribution was uneven, a mass was seen in the right posterior lobe of the liver, the size was about 13.0 × 9.87 cm, the shape was oval, the interior was hyperechoic, the distribution was inhomogeneous, the edges were clear, the intrahepatic ductal structures were displaced by compression. (b) Color Doppler ultrasonography showed that blood flow signal was visible within and around the mass, and pulsed Doppler showed that the blood flow was with high velocity and high resistance with RI 0.87.

**Figure 2:** CT scan showed a round-like slightly hypointense shadow in the right lobe of the liver with poorly defined borders; enhancement scan showed significant enhancement in the arterial phase and relative hypointensity in the portal vein phase and delayed phase, with a continuous decrease in the degree of enhancement and a “fast showing and fast-out” enhancement.

**Table 1:** General characteristics of 98 HCC patients and 50 patients with benign liver lesions.

Characteristics		Study group (98 cases)	Control group (50 cases)
Gender	Male	59	32
	Female	39	18

Age		57.32 ± 6.81	55.67 ± 8.42

Clinical stage	Stage I	18	
	Stage II	47	
	Stage III	24	
	Stage IV	9	

Degree of differentiation	Highly differentiated	37	
	Moderately differentiated	26	
	Lowly differentiated	20	
	Undifferentiated	15	

Disease type	Hepatitis pseudotumor		5
	Hepatic hemangioma		9
	Cirrhotic hyperplastic nodules		23
	Hepatic granuloma		13

**Table 2:** Comparison of blood flow parameters between the hepatocellular carcinoma group and benign control group.

Group	Cases	Diameter of hepatic artery (mm)	Hepatic artery peak velocity (cm/s)	Minimum hepatic artery flow rate (cm/s)	RI	Portal vein flow velocity (cm/s)
HCC group	98	5.6 ± 0.4e	119.22 ± 16.34e	22.86 ± 2.69^a^	0.85 ± 0.07^a^	10.53 ± 1.02^a^
Control group	50	4.1 ± 0.3	61.24 ± 6.59	8.37 ± 1.32	0.43 ± 0.03	17.51 ± 3.64
t		3.286	7.369	3.698	4.365	3.204
P		0.017	<0.001	0.012	0.006	0.023

^a^ *P* < 0.05, compared with the control group.

**Table 3:** Comparison between the results of color Doppler ultrasonography, CT, and serum AFP in the diagnosis of hepatocellular carcinoma and pathological diagnosis (*n*).

		Pathological diagnosis	
		Malignancy	Benign
Color Doppler ultrasonography	Malignancy	78	4
	Benign	20	46

CT	Malignancy	84	5
	Benign	14	45

AFP	Malignancy	65	5
	Benign	33	45

Combined examination	Malignancy	95	6
	Benign	3	44

**Table 4:** Comparison of the value of color Doppler ultrasonography, CT, and serum AFP alone and in combination in the diagnosis of hepatocellular carcinoma (% (*n*)).

	Sensibility	Specificity	Accuracy	Positive predictive value	Negative predictive value
Color Doppler ultrasonography	79.59 (78/98)	92.00 (46/50)	83.78 (124/148)	95.12 (78/82)	69.70 (46/66)
CT	85.71 (84/98)	90.00 (45/50)	87.16 (129/148)	94.38 (84/89)	76.27 (45/59)
AFP	66.33 (65/98)	90.00 (45/50)	74.32 (110/148)	92.86 (65/70)	57.69 (45/78)
Combined examination	96.94 (95/98)	88.00 (44/50)	93.92 (139/148)	94.06 (95/101)	93.62 (44/47)
X^2^	33.626	0.444	22.904	0.363	19.522
*P* value	<0.001	0.931	<0.001	0.948	<0.001

Compared to single tests, *p* < 0.05.

## Data Availability

The data to support the findings of this study are available on reasonable request from the corresponding author.
